# Enterprise Information Security Management Using Internet of Things Combined with Artificial Intelligence Technology

**DOI:** 10.1155/2022/7138515

**Published:** 2022-06-14

**Authors:** Hongbin Sun, Shizhen Bai

**Affiliations:** School of Management, Harbin University of Commerce, Harbin 150028, Heilongjiang, China

## Abstract

This work is conducted to deal with the information security of enterprise management under the background of current global informatization, popularize the modern Internet of Things (IoT) management technology of enterprises, and maintain the information security of enterprises and provide modern upgrading means for enterprise management. In this work, it firstly introduces the application scenarios of current Internet and Artificial Intelligence (AI) technology and expounds the IoT technology. Secondly, the enterprise management platform is designed, the requirements of enterprise modern management are analyzed, and then the design requirements of system functions and the design of the information security architecture of the IoT are proposed. Furthermore, an enterprise information security management platform is designed, which covers four parts: IoT data mining management, equipment management, key management, and database management. In addition, the performance of the security management platform is tested from four parts: concurrency testing, stress testing, large data volume testing, and security testing. The research results show that the IoT-based enterprise information security management platform designed in this work under the background of AI has perfect functions and stable performance of each module. Concurrency testing, stress testing, large data volume testing, and stability testing are performed on it, and the success rate of the platform in each task reaches 100%. The average response time of concurrent testing and stress testing is about 0.13 seconds, and that of the event entry events is 0.25 seconds. The central processing unit (CPU) occupancy rate in each monitoring task is always lower than 20%. Therefore, it is determined that the performance of the IoT-based enterprise information security management platform designed in this work is sufficient to meet the daily management of enterprises. This work can provide a guarantee for enterprise information security management using AI technology, setting an example for future related research.

## 1. Introduction

With the continuous improvement of living standard and technological level, artificial intelligence (AI) gradually enters people's life. Internet information technology is also widely applied in social production and life and human society fully enters informatization age [1–3]. Internet of Things (IoT) is another wave in information industry following computers, Internet, and mobile communication network [4]. Everything in the world, including small things such as watches and keys and big objects such as vehicles and buildings, can become intelligent by embedding a tiny sensor chip and it can “automatically speak.” Based on wireless network technology, people can “talk” with objects. Besides, objects can “communicate” with each other, which is called IoT [5–7]. In China, it is also called sensor network. The sensor network refers to a huge network formed by combining various information sensor equipment and Internet. The construction of IoT depends on physical signal sensor, radio frequency identification (RFID) [8], and global positioning system (GPS) [9] to acquire target information in real time. After that, it realizes the connection between the target and the network and then achieves the interconnection among everything and intelligent recognition and management of the interconnection between human and things, which is the extension and expansion of Internet technology [10–12].

IoT technology has a profound influence on people's production and life, while causes information security problems to people's life.

The IoT needs to identify the user's identity when using it, which has become an inherent leak vulnerability, and it is difficult to solve it from the perspective of technical means. With the increasingly powerful functions of the applied smart devices, the boundaries between the IoT network and the physical life of human beings are constantly blurred. This has led to a series of technical ethical issues and security issues, which mainly focus on the need to obtain user data and privacy when using the IoT. In addition, it becomes particularly sensitive when it comes to enterprise information security.

AI is a new technical science that explores and develops theories, methods, technologies, and application systems for simulating, extending, and expanding human intelligence. AI is a branch of computer science that attempts to understand the essence of intelligence and produce a new kind of intelligent machine that can respond in a similar way to human intelligence. Research in this field includes robotics, language recognition, image recognition, natural language processing, and expert systems. By automating routine tasks, robots can take on tasks related to analysis, fine-tuning, and problem solving. Therefore, applying AI at work will reduce the workload, give humans the ability to improve their skills, and free them from monotonous work, so that employees can focus on the creativity of their work. The use of AI techniques in hazardous tasks will reduce human safety risks [13].

The IoT has brought changes to the mode of human life and penetrated into all aspects of human life, but it has also brought about information security, which leads to a series of technical ethical and security issues. These issues mainly focus on the need to obtain user data and privacy when the IoT is applied, which becomes particularly sensitive when it comes to enterprise information security.

IoT facilitates several advantages in everyday life in the business sector. Some of its advantages are as follows. Firstly, it realizes efficient resource utilization: if how each device functions and works can be understood fully, it can definitely improve the efficient utilization of resources and monitor natural resources. Secondly, it minimizes human labor: when IoT devices interact and communicate with each other and complete a large number of tasks, they can minimize human labor. Thirdly, it can save time: because it reduces manpower, it definitely saves time. Time is a major factor that can be saved through IoT platforms; the new digital technology transformation of IoT with AI and cloud network storage provides accuracy, storage facilities, and accessibility anytime and anywhere. Fourthly, it enhances data collection: network and collecting relevant data. Finally, it improves security: if the system can connect all of these things to each other, then it can make the system more secure and efficient. The shortcomings of IoT also present a series of significant challenges. Some of the disadvantages of IoT are given below. *a*. Security: IoT systems are interconnected and communicate through the network. Despite any security measures, the system provides almost no control and can initiate various cyberattacks. *b*. Privacy: even without actively participating users, IoT systems can provide the most detailed and extensive personal data. *c*. Complexity: designing, developing, maintaining, and supporting large technology-to-IoT systems are quite complex [14].

Singh et al. (2021) proposed a comprehensive cybersecurity framework that can effectively establish a target security environment. The framework has two structural dimensions and two program dimensions. Structural dimensions include scope and evaluation criteria; and the program dimensions include process and assessment tools. The framework uses a comprehensive strategy technology organization people environment (STOPE) view; and its evaluation criteria are considered open to a variety of criteria. For the procedural dimension, the framework uses a define-measure-analyze-improve-control (DMAIC) cycle to advance the process, and the framework considers the use of various assessment tools [15]. Zuo et al. (2020) proposed a comprehensive information security evaluation model based on multilevel decomposition feedback. The evaluation model provided ideas for the evaluation of IoT information security and guided security decision makers for dynamic protection. Firstly, an overall evaluation index system is established in this work. It includes four main contents (threat information indicators, asset indicators, vulnerability indicators, and management indicators). In addition, it covers 10 secondary indicators and service continuity such as system protection rate, attack detection rate, confidentiality, availability, controllability, identifiability, number of vulnerabilities, vulnerability hazard level, personnel organization, and enterprise classification [16]. Using discrete event modeling, Durowoju et al. (2020) explored the impact of disruptions caused by information security breaches on supply chain performance and the externalities of partial integration on nonparticipants and explored the impacts of breach disruption frequency and remediation length on supply chain performance [17]. To sum up, previous researches mainly focus on detecting and finding vulnerabilities in security threat frameworks. The innovations of this work are to design an enterprise information security management platform covering four parts: IoT data mining management, equipment management, key management, and database management, and improve and reorganize the original physical security framework in four aspects: concurrency testing, stress testing, large data volume testing, and security testing. The objective of this work is to provide new ideas for the application of information security technology in the modern management of enterprise based on the IoT and to provide a new perspective for promoting the IoT in industrial and commercial management in the future.

In today's information society, various new computer technologies emerge in an endless stream. As a result, the IoT information management technology applied to the modern management of enterprises has been born. Based on the IoT technology and AI technology, an enterprise management platform on information security is designed to achieve the real-time, efficient, and accurate management of enterprise information. It aims to provide new idea for the application of information security technology in enterprise management.

## 2. Design of Enterprise Management Platform

### 2.1. Demand Analysis of the Management Platform

The enterprise management platform on IoT information security has to meet the current modern management needs, and its overall main functions are shown in Figure 1 below.

The functions of the management platform to be achieved include authorization and revocation, employee scheduling, data storage and backup, rank role management, and data encryption and mining [18, 19]. Its functions are shown in Table 1 below.

### 2.2. System Function Design

#### 2.2.1. IoT

IoT is the Internet connecting everything, which contains two meanings.

- The core and foundation of IoT is Internet, and IoT is the extended and expanded network based on Internet.
- It realizes the information exchange and communication between objects, which is the interdependence of things. Based on intelligence, recognition technology, pervasive computing, and other communication awareness technologies, IoT is widely applied in network convergence. Therefore, it is also called the third wave of the development of global information industry after computers and Internet. IoT is the expansion of the application of Internet, which is not so much a network as business and applications. Hence, application innovation is the core of IoT development. User experience-centered innovation is the soul of IoT development [20].

The framework of IoT is divided into three layers, including perception layer, network layer, and application layer.

The difference between IoT and traditional Internet is that the former one is the wide application of various perception technologies. A large number of multiple types of sensors are deployed on IoT and each of them is an information source. The content and format of the information captured by different sensors are different. The data obtained by sensors is real time. Sensors periodically collect environmental information at certain frequency and update data constantly. Hence, it is a pervasive network constructed on Internet. The essential foundation and core of IoT technology are still Internet. It is integrated with Internet through various wired and wireless networks to transmit object information accurately in real time. The information acquired regularly by the sensors on IoT needs to be transmitted through the network. Because of its huge number, numerous information is generated. In the process of the transmission, the data must adapt to a variety of heterogeneous networks and protocols to ensure the accuracy and timeliness of data.

IoT not only offers sensor connectivity, but also possesses the capacity of intelligent processing. It can perform the intelligent control over objects. Besides, it combines sensors with intelligent processing and utilizes cloud computing, pattern recognition, and other various intelligent technologies to its application fields. Meaning data are analyzed and processed from the massive data obtained by sensors to adapt to the various needs of different users and find new application fields and patterns. The spiritual essence of IoT is to offer the free interaction between application scenario and users not constrained to any occasion and time. It relies on cloud service platform and interconnecting embedded processing software to pay less attention to technologies, strengthen the positive interaction with users, and offer better user experience. In addition, the timelier data acquisition and suggestion analysis as well as freer work and life are the physical supports to intelligent life [21].

RFID of IoT is applied in the research.  Figure 2 displays the basic model of radio frequency identification system below. Electronic tags are also called radio frequency tags, transponders, and data carriers. Readers are also called reading devices, scanners, communicators, and readers (the selection of the name of readers depends on whether electronic tags can rewrite data wirelessly). The spatial (contactless) coupling of radio frequency signals between electronic tags and readers is achieved by coupling elements. Within coupling channels, energy transmission and data exchange are realized according to sequential relationship.

After the tags enter magnetic fields, the radio frequency signals emitted by receiving readers send the product information stored in chips by the data obtained by induction current. Alternatively, the tags actively send a frequency signal. The current application of RFID technology mainly refers to RFID tags. The electronic tag of each object has a unique ID for the query of the digital information about the corresponding objects. Hence, the core of RFID system is electronic tag, which contains a chip and an antenna. The function of chip is the preprocessing of the electronic signals it receives and the transmission of ID information to the card reader. The function of the antenna is receiving and sending signals [22–24].  Figure 3 shows the general structure of tag chip below.

Card reader is used for reading and writing RFID tags. The reader sends radio frequency signals with certain frequency through transmitting antenna. When electronic tags enter the working area of transmitting antenna, induction current is generated and the tags obtain energy to be activated. The tags send their own codes and other information by card built-in transmitting antenna. After that, the system receiving antenna receives the carrier signals sent from the tags and then transmits them to the reader through the antenna regulator. Next, the reader demodulates and decodes the signals it receives and then transmits them to the background main system for relevant processing [25].  Figure 4 presents its internal structure below.

RFID system can own one or multiple card readers. It can perform data processing, data exchange, data management, data transmission, and communication with the help of the upper layer of computer system.

Based on traditional positioning algorithm, Landmarc algorithm is proposed. The core idea of the algorithm is the construction of centroid weight algorithm based on received signal strength indicator (RSSI). Based on the real-time acquisition of RSSI of reference tags and the tags to be positioned, *n* reference tags closest to RSSI of the tags to be positioned are selected. After that, the weights of *n* reference points are calculated according to the similarity of RSSI. In addition, the position of the tags to be positioned is weighted and estimated. Because Landmarc algorithm can obtain RSSI in real time, it can automatically adapt to environmental changes to realize more accurate and reliable positioning. Two antennas face the tag array. One is aligned with the left boundary of the tag array, and the other is aligned with the right boundary. After one scan, the two antennas acquire RSSI of each tag. As a result, each tag has two RSSI, which are labeled as (RSSI-1, RSSI-2). RSSI-i refers to the RSSI obtained by i^th^ antenna. T7 represents the tag to be positioned and the rest are reference tags. According to (RSSI-1, RSSI-2) of each tag, the distance between T7 and other tags is calculated. Besides, 4 tags with the shorter distance from T7 are selected as the adjacent tags. Finally, the coordinates of the adjacent tags are used for the inverse distance weighed voting to estimate the coordinate of T7 [26, 27].

The basic Landmarc algorithm is as follows.

(a) RSSI of the tag to be positioned is read and recorded as *S*=(*S*_1_,*S*_2_). *S*_*i*_ refers to RSSI of the tag obtained by antenna *i*. RSSI of the reference tag is read and expressed as *θ*_*j*_=(*θ*_*j*1_,*θ*_*j*2_). *J* denotes the j^th^ reference tag and *θ*_*j*_ refers to RSSI of reference tag *j*.
(b) Euclidean distance between the tag to be positioned and reference tag is calculated, as expressed by (1) below.
  (1) $$\begin{array}{c} E_{j}=\sqrt{{\left(S_{1}-\theta_{j1}\right)}^{2}+{\left(S_{2}-\theta_{j2}\right)}^{2}}. \end{array}$$
In (1), *E*_*j*_ represents the position relationship between the tag to be positioned and reference tag. Smaller values of the two tags indicate the shorter distance between them.
(c) A total of 19 reference tags *E*=(*E*_1_,...,*E*_19_) are obtained. *d. E*_*j*_ is compared to select 4 smallest reference tags. *e*. The weights of 4 closest reference points are calculated, as shown in (2). *W*_*j*_ refers to the weight of the closest reference point *j*.
  (2) $$\begin{array}{c} W_{j}=\frac{1/E_{j}^{2}}{\sum_{i=1}^{4}1/E_{j}^{2}}. \end{array}$$
(d) The coordinate of the tag to be positioned (*x*',*y*') is estimated, as shown in equation (3). (*x*_*i*_,*y*_*i*_) is the known coordinate of reference point.
  (3) $$\begin{array}{c} \left(x{}^{\prime },y{}^{\prime }\right)=\sum_{i=1}^{4}w_{i}\left(x_{i},y_{i}\right). \end{array}$$
(e) The positioning accuracy is assessed, as shown in (4) below. (*x*,*y*) represents the real coordinate of the tag to be positioned.
  (4) $$\begin{array}{c} e=\sqrt{{\left(x-x{}^{\prime }\right)}^{2}+{\left(y-y{}^{\prime }\right)}^{2}}. \end{array}$$

#### 2.2.2. IoT Security Architecture Design

The IoT network module is divided into four modules: application layer, processing layer, transmission layer, and perception layer.  Figure 5 below shows its security architecture, and the role of each module is shown in Table 2 below.

The enterprise management platform on information security is built using Python for programming and development. The platform contains three layers: application layer, communication layer, and perception layer. The management system includes management of hardware, system, data mining process and results, encryption, system and information security, and data services. The communication layer is used for data transmission, including various network connection methods. In addition, the perception layer consists of various sensors [28].

#### 2.2.3. AI Technology

AI is a theory, method, technology, and application system that uses digital computers or machines controlled by digital computers to simulate, extend, and expand human intelligence, perceive the environment, acquire knowledge, and use knowledge to obtain the best results. The core idea of AI is to construct intelligent artificial systems. AI is a knowledge project that uses machines to imitate human beings to complete a series of actions to achieve functions similar to human understanding, thinking, reasoning, and problem solving.

The core technologies of AI mainly include deep learning, computer vision, natural language processing, and data mining [29]. Machine learning is a technology analyzing how computers simulate or realize the learning behavior of animals in order to learn new knowledge or skills, rewrite existing data structures, and then improve program performance. From a statistical point of view, it is to predict the distribution of data, learn a model from the data, and then use this model to predict new data. This requires that the test data and training data must be the same distribution. Its basic feature is an attempt to mimic the pattern of information transmission and processing between neurons in the brain. The most notable applications are in the fields of computer vision and natural language processing. Obviously, “deep learning” is strongly related to “neural network” in machine learning, and “neural network” is also its main algorithm and means; or the “deep learning” can be called as an “improved version of neural network” algorithm. The main idea of deep learning is to simulate human neurons. Each neuron receives information and transmits it to all adjacent neurons after processing. The following are several commonly used artificial intelligence technology application areas.

- Natural language generation: AI speaks (or writes) the correct word, which can coherently express an accurate meaning and can be easily understood. It is very difficult for an AI that processes information in a completely different way from the human brain.
- Voice recognition: it can convert human speech into a language suitable for computer recognition, so it is currently used in interactive voice response systems and mobile applications. Every day, more and more systems transcribe and convert human language into a language suitable for computer recognition.
- Machine Learning: computers can learn, and they can be very smart. Machine Learning is a discipline of computer science and a branch of AI. Its goal is to develop technologies that allow computers to learn. Machine Learning platforms are gaining more and more attention every day by providing algorithms, application programming interfaces (APIs), development and training tools, big data, applications (APPs), and other machine AI.
- Virtual Agents: it is undeniable that Virtual Agents or “Chatbots” (or “bots” for short) are also experiencing a huge renaissance with the rapid development of innovation and technology. They are currently used in customer service and service support, and they are used as smart home stewards. Some companies that provide Virtual Agents include Amazon, Apple, various smart speakers, Google, International Business Machine (IBM), IPsoft, and Microsoft.
- Decision management: intelligent machines are able to introduce rules and logic into AI systems and can be used for initial setup/training, ongoing maintenance, and tuning. It is used in a wide variety of enterprise applications to aid or execute automated decision-making. Companies are investing heavily in hardware design for machine learning and AI to dramatically accelerate the development of next-generation applications. Graphics Processing Units (GPUs) and specially designed equipment efficiently run the computational work of AI. Some companies that focus on human-optimized hardware are Google, IBM, Intel, and Nvidia.
- Deep Learning platforms: Deep Learning is the fastest growing field and the biggest trend in machine learning. A set of artificial neural networks (ANNs) has multiple levels of learning algorithms and corresponds to different levels of abstraction. Some applications of deep learning, like automatic speech recognition, image recognition, optical character recognition, and natural language processing, can classify/categorize/predict any entity to be perceived and digitized.
- Robotic process automation: process automation in the enterprise is possible because scripts and algorithms can simulate and automate human tasks to support enterprise processes. Robotic process automation is applied for specific jobs or tasks where hiring labor is too costly or inefficient.
- Text analysis and natural language processing: natural language processing is concerned with the interaction between computers and human (natural) language. The technology utilizes text analysis techniques and applies statistical methods and machine learning to understand the structure of sentences as well as their meaning and intent. They are also used for automation of huge amounts of data and applications to extract unstructured data.
- Biostatistics: this group of techniques is used to identify, measure, and analyze aspects of human body structure, morphology, and behavior. It allows for more natural interactions between humans and machines, including those related to touch, image, language, and body language recognition.

Deep Learning is a new research direction in the field of machine learning, which is introduced into machine learning to make it closer to the original goal, AI. The most notable applications of deep learning are in computer vision and natural language processing. Each neuron receives information and transmits it to all adjacent neurons after processing. Deep Learning is to learn the inherent laws and representation levels of sample data, and the information obtained during these learning processes is of great help to the interpretation of data such as text, images, and sounds. Its ultimate goal is to enable machines to have the ability to analyze and learn like humans and to recognize data such as words, images, and sounds. Deep Learning is a complex machine learning algorithm that has achieved results in speech and image recognition far exceeding previous related technologies. Deep Learning has achieved many results in search technology, data mining, machine learning, machine translation, natural language processing, multimedia learning, speech, recommendation, and personalization technology. Deep Learning enables machines to imitate human activities such as audio-visual and thinking, solves many complex pattern recognition problems, and makes great progress in AI-related technologies. In this work, the deep learning techniques are adopted to construct the dataset to train the model.

#### 2.2.4. System Function Design

The key functions of the system include four parts: IoT data mining management, equipment management, key management, and database management.

*(1). IoT Data Mining*: it includes functions such as data collection, data filtering, data mining, and result display. To build an information collection system, data mining has to be performed to find the data that is helpful for model building in the massive data and form the data set needed for model training.  Figure 6 below shows the complete steps of data mining.

Data mining technology is the application of machine learning technology to discover relevant data in massive data. Data prescreening, mid-stage processing, and postdata transformation have obvious effects on data processing results. The technologies and functions that need to be applied in the data mining process are to collect a large amount of data. In order to ensure that the number of data applications in the later stage is sufficient, it is necessary to collect comprehensive data as much as possible. There are mainly missing values, outliers, deduplication, and noise data processing to deal with the missing data selection caused by accidental errors in the previous step. Data mapping processing is divided into three situations: text encoding conversion, format conversion, and numerical mathematical processing. The sensor is expressed as *w*={*w*_1_, *w*_2_,…, *w*_*n*_}. When the data collected by different sensors at different times *t* is expressed as numerical data *D*={*w*_1_*t*1__, *w*_2_*t*2__,…, *w*_*n*_*tn*__} for mathematical processing, (5) can be used for numerical conversion for observation if a certain value changes exponentially, while it is processed in the form given in (6) when the numerical data is in the form of a power function [30].

(5) $$\begin{array}{c} f\left(t\right)={\text{log}}_{n}\left(t+k\right), \end{array}$$

(6) $$\begin{array}{c} f\left(t\right)=\sqrt[{n}]{t}. \end{array}$$

*f(t)* is the converted data, *n* is the coding serial number, *t* represents the value before conversion, and *k* refers to a constant given by the system. In the process of data conversion, the data is stored in multiple systems. If the subsequent processing needs to be operated in multiple systems, errors will occur and the process will be doubled. Therefore, it is necessary to integrate and summarize the data into a database.

*(2) Data Analysis.* It is to analyze the relationship between the sample data and search for the laws hidden in the data. There are generally two methods as follows: Pearson correlation coefficient (PCC) and logistic regression analysis. PCC is used to measure the linear correlation between two variables and is often used to measure the correlation and size. Its equation is as follows:

(7) $$\begin{array}{c} \rho \left(x,y\right)=\frac{\mathrm{cov}\left(X,Y\right)}{\sigma_{X}\sigma_{Y}}\\ =\frac{E\left(X-\mu x\right)\left(Y-\mu y\right)}{\sigma_{X}\sigma_{Y}}. \end{array}$$

Its value range is between [−1, 1]. When it is less than 0, negative correlation is found; when it is greater than 0, positive correlation is found; when the absolute value of correlation is less than 0.09, there is no correlation. When the absolute value of the correlation is between 0.1 and 0.3, the correlation is weak; when the absolute value of the correlation is between 0.3 and 0.5, the correlation is medium; and when the absolute value of the correlation is between 0.5 and 1.0, the correlation is strong. *ρ* is the overall correlation coefficient, *cov(X,Y)* represents the covariance between the samples *X* and *Y*; *σ*_*X*_ and *σ*_*Y*_ represent the sample standard deviation of the samples *X* and *Y*, respectively; *E* is the sample expectation, and *μ* refers to the sample mean.

(8) $$\begin{array}{c} r=\frac{\sum_{i=1}^{n}\left(X_{i}-\bar{X}\right)\left(Y_{i}-\bar{Y}\right)}{\sqrt{\sum_{i=1}^{n}{\left(X_{i}-\bar{X}\right)}^{2}}\sqrt{\sum_{i=1}^{n}{\left(Y_{i}-\bar{Y}\right)}^{2}}},\\ r=\frac{1}{n-1}\left(\sum_{i=1}^{n}\frac{X_{i}-\bar{X}}{\sigma_{X}}\right)\left(\frac{Y_{i}-\bar{Y}}{\sigma_{Y}}\right). \end{array}$$

In the above equations, *r* is the Pearson correlation coefficient; *X*_*i*_ and *Y*_*i*_ are the data value of the numbered sample *i*, $\bar{X}$ is the sample mean, and *σ* refers to the sample standard deviation.

Logistics regression analysis is used to represent each influence relationship of multiple influencing factors. The calculation equations are shown in (9) and (10) below

(9) $$\begin{array}{c} f\left(x\right)=\frac{1}{1+\exp\left(-x-\mu /\gamma \right)}, \end{array}$$

(10) $$\begin{array}{c} f\prime \left(x\right)=\frac{\exp\left(-x+\mu /\gamma \right)}{\gamma 1+\exp\;{\left(-x+\mu /\gamma \right)}^{2}}. \end{array}$$

*f(x)* represents the distribution function of the sample set *X*, and *f'(x)* is the density function of the sample set *X*. At this time, *x* obeys the logistic regression distribution.

*(3) Hardware Management*. It is designed according to the three-tier architecture, and its functional structure is shown in Figure 7 below.

Due to the huge amount of hardware in the management system, the function of the hardware management function module must be relatively powerful, so a three-tier structure and more components are set up.

*(4) Key Management*. Its role is to ensure the security of data transmission, which is different from mainstream encryption methods: the encryption method of the IoT will make memory allocation very tight. Therefore, the wireless sensor network (WSN) key predistribution algorithm based on regular hexagon deployment is selected.

*(5) Database Design.* An open source relational database management system is chosen to store data, so as to improve the versatility. The data tables contain equipment information tables, security information tables, etc. [31].

#### 2.2.5. The Overall System Architecture

The platform adopts the most popular Browser/Server (B/S) structure. The most obvious advantage of the B/S structure is that the client configuration requirements are very low. As long as you have a computer with a browser installed and access the network, you can use the system. Secondly, the maintenance cost of the B/S structure is also very low. During the upgrade, the client can see the latest system immediately as long as the upgrade is performed on the server side, and there is no need to upgrade each client, which greatly reduces the time cost. In addition, JavaFramework is selected as the development framework in the B/S structure.

Advantages of JavaFramework are summarized as follows. JavaFramework is designed based on the three-tier architecture of Struts, so it has all the advantages of Struts. In addition, a lot of custom tags are developed on top of it. In order to facilitate the code writing of developers, these custom tags cover many aspects such as public functions, permission control, and automatic code generation. These custom tags not only standardize the code writing of developers, but also optimize the efficiency and security of the code to a great extent. In this case, developers only need to concentrate on the business logic of the system when completing the code, without having to consider other factors.  Figure 8 below shows the overall structure of the system.

The main functional modules of this platform are as follows. *a*. Organization and workflow engine module: it sets up the organizational departments of large enterprises and various units, sets user personnel permissions, and configures the workflow engine to support business process flow. *b*. IoT data module: large enterprises and various units manage the unit information, information systems, and information asset information of each unit, realizing the filling and reporting function of basic information security data of each unit. *c*. Level protection management module: it is a platform for large enterprises and various units to carry out level protection management work, including system rating, filing, self-assessment, and evaluation management. *d*. Risk management module: it refers to a management of information security risk assessment process of large enterprises and various units, including risk identification, assessment, disposal, reporting, and other processes. *e*. Security incident reporting module: it is to give the security incident reporting process of large enterprises and various units, including incident reporting, incident grading, incident investigation and analysis, and rectification. *f*. Emergency response module: it is responsible for emergency plan management of large enterprises and various units, emergency drill information management, emergency result feedback, etc. *g*. Rectification planning module: it is responsible for the tracking management function of large enterprises and various units for information security rectification work. *h*. Security inspection module: it refers to the process management for large enterprises and various units to carry out information security inspection work.

#### 2.2.6. The System Function Module Design

*a*. Basic data includes unit information, information system, and information asset information managed by large enterprises and subordinate units, realizing the filling and reporting function of information security basic data of each unit. The basic data that needs to be filled in include information system name, serial number, system carrying business, system service, system-related data, host storage device, network/security device, business application software, and security management personnel. *b*. The functional module of graded protection management is to support large enterprises and subordinate units to carry out graded protection management of information security of important information systems in accordance with relevant policy standards for graded protection, including data collection, grading, filing, self-inspection, rectification, and evaluation of information systems of each unit and other related work activities. There are built-in graded protection standard rules and related knowledge and experience for the platform, which provides effective support for the data reporting and analysis process. By summarizing the data, the basic situation of graded protection related work of each unit can be statistically analyzed, and the security status can be compared by year and unit. *c*. Risk management module. *d*. Security incident notification module. *e*. Emergency response module. *f*. Revise the planning function module. *g*. Security check module.

#### 2.2.7. Key Predistribution Algorithm

In a large-scale wireless sensor network, nodes communicate with each other in the way of data multihop. It is required that any node can independently establish a communication key with surrounding nodes to ensure the security and integrity of data. However, it is impossible to use traditional methods to complete under the current bandwidth conditions of sensor networks, especially in large-scale networks. Random predistribution key mechanism: at the cost of a certain storage consumption, a secure link is established through optimization in three stages: key predistribution, link establishment, and link update. Any node only needs to exchange data with its surrounding nodes to complete the key negotiation, which minimizes the bandwidth and energy consumption caused by data transmission and becomes a better solution. Therefore, the Real-time Kernel Protection (RKP) is undertaken as the random predistributed key algorithm in this work.

#### 2.2.8. System Test

The following test environment architecture is constructed using Python as the development language, the test hardware environment is a web application server, and a computer terminal server is configured with one 8-core central processing unit (CPU), one 1 TB hard disk, a 16G memory card, and two GE network cards. The operating system is Windows7, the application software is Apache Tomcat 6.0, and the test software is LoadRunner9.5 and IE browser. 400 virtual computer terminals and web servers are constructed for the performance test; 400 virtual users are set, and each user is arranged with a different IP address and uses his own account to log in to collect information. 1000 groups of user data are collected to construct a dataset, of which 800 groups are made into training sets and 200 groups are made into test sets to train the model.

## 3. Results

### 3.1. Version Test Results

The version test of the constructed enterprise management platform of modern IoT information security is carried out, and the test results are shown in Table 3 below.

Table 3 above suggests that seven items of the management platform are tested. The test started in early September 2021 and ended in early October. During this period, the sensor data collection effect, data protection capability, data security test, data security log, security risk assessment, system internal correction, and system authorization management have been tested, and the test results are all passed. Therefore, the platform performs well in version test performance.

### 3.2. Performance Test Results

The performance is tested from four aspects: concurrency testing, stress testing, large data volume testing, and security testing. The results are shown in Figure 9 below.

As shown in the figure above, in the concurrent experiment, the average response time of information input, gap analysis, and event entry is 0.136s, 0.137s, and 0.138s, respectively. In the stress test, the average response time of information input, gap analysis, and event entry is 0.140s, 0.146s, and 0.137s, respectively. In the big data test, the average response time of information input, gap analysis, and event entry is 0.142s, 0.126s, and 0.251s, respectively. In the security test, the average response time of information input, gap analysis, and event entry is 0.146s, 0.124s, and 0.250s, respectively. Among the average response times of these four tests, the average response time of concurrent experiments and stress tests is about 0.13 seconds, while the average response time of event entry is 0.25 seconds in the big data test and stability test, which indicates the strong feedback ability of the system.

As shown in the figure above, the CPU utilization rate in application server monitoring and database server monitoring has always been lower than 20%. The CPU utilization rate of the information input, gap analysis, and event entry in the concurrency test is 36.1%, 13.9%, and 26.2%, respectively. The CPU utilization rate of the information input, gap analysis, and event entry in the stress test is 36.4%, 13.7%, and 26.1%, respectively. The CPU utilization rate of the information input, gap analysis, and event entry in the large data volume test is 36.3%, 13.8%, and 26.3%, respectively. The CPU utilization rate of the information input, gap analysis, and event entry in the security test is 13.7%, 26.0%, and 14.1%, respectively. Such results suggest that the algorithm and operating structure of this platform are relatively simple, and the demand for CPU is not high.

For memory utilization rate, the storage spaces for information input, gap analysis, and event entry in the concurrent test are 5426B, 6213B, and 2681B, respectively. The storage spaces of the information input, gap analysis, and event entry in the stress test are 5437B, 6225B, and 2692B, respectively. The storage spaces of information input, gap analysis, and event entry in the large data volume test are 5417B, 6198B, and 2654B, respectively. The storage spaces of information input, gap analysis, and event entry in the security test are 6242B, 2673B, and 6186B, respectively. The use of information entry and gap analysis is below 6 GB, the use of event entry is below 7 GB, and the transaction success rate obtained from the test is 100%, indicating that it will be completed. This shows that the IoT-based enterprise information security management platform designed in this work is reasonable.

## 4. Conclusion

In this work, an IoT-based modern enterprise information security management platform is designed. Firstly, the development status of AI technology is analyzed, and the operation principle of the IoT and the collection, transmission, and preservation of data information are analyzed. Secondly, a modern enterprise information security management system is designed by analyzing the information security requirements of modern enterprises. Finally, the performance test of this work platform is carried out, and the version test and performance test results of the platform are obtained. The final practical application results show that the test results of the enterprise modern management system for IoT information security proposed in this work are all qualified under the background of artificial intelligence; the average response time to an event is less than 0.25s, the CPU usage does not exceed 20%, and the memory requirement is not large. Therefore, the system constructed in this work has a better effect on enterprise information security management.

Although it basically achieves the original expected research objectives, some valuable research conclusions are also obtained. However, there are still many deficiencies in the research work, and the research conclusions are limited by the following two factors. (1) The information security needs of enterprises in different industries are not explored. (2) The current management platform has a high demand for memory. This also points the way for our future research. In the future, it will focus on two aspects. (1) It should consider the different needs of enterprises in different industries for information security. (2) It should further increase the collection of various enterprise information security data and improve the algorithm to reduce the system's demand for memory.

## Figures and Tables

**Figure 1:** Main functional parts of the platform.

**Figure 2:** Schematic diagram of the basic structure of the RFID system.

**Figure 3:** General structure of tag chip.

**Figure 4:** Internal structure of card reader.

**Figure 5:** IoT network security architecture.

**Figure 6:** Complete steps of data mining.

**Figure 7:** The three-tier architecture of hardware management.

**Figure 8:** Overall structure of the system.

**Figure 9:** (a) Average response time. (b) Application server processor utilization. (c) Database server processor utilization. (d) Application server memory usage. (e) Database server memory usage.

**Algorithm 1:** Internet of Things-Based Enterprise Modernization Management BP-PSO Algorithm

**Table 1:** Functional requirements of the management system.

Serial number	Type of function	Function descriptions
1	Authorization and revocation	It can add permission information, view permission information, delete permission information, and replace permission information.
2	Employee scheduling	It can realize employee information entry, employee information cleaning, employee information viewing, and employee information modification.
3	Data storage and backup	It can realize data storage and transfer, data upload to the cloud, data download, and system database restoration.
4	Rank role management	It can manage enterprise roles.
5	Data encryption and mining	It can realize data encryption using encryption algorithms, including collecting data, filtering data, mining data information, and drawing conclusions.

**Table 2:** The role of each module.

Serial number	Name	Composition	Effect
1	Perception layer	Wireless sensor	It is a part of the bottom layer, which controls physical security and is used to ensure the integrity of IoT information collection data and not be destroyed or stolen.
2	Information collection layer	Information collector	Its information security needs to be managed to prevent the data collection process from being used and controlled, and the technology of the perception layer is encrypted with key management and chip design.
3	Information transmission security layer	Hard disk	Data transmission ensures the smooth collection of data and cooperates with security management technologies, such as wireless network security, routing security, firewall, and virtual network technology.
4	Information processing layer	Hard disk	It is to ensure the security of information processing and storage. It is composed of cloud storage and security management. Its technologies include analysis of security data, viruses, monitoring data, and data mining results.

**Table 3:** Version test results.

Serial number	Start time	End time	Tested item	Test results
1	2021.9.7	2021.9.12	Sensor data collection	Qualified
2	2021.9.13	2021.9.17	Data protection capability	Qualified
3	2021.9.18	2021.9.23	Data security testing	Qualified
4	2021.9.24	2021.9.29	Data security log	Qualified
5	2021.9.30	2021.10.1	Security risk assessment	Qualified
6	2021.10.2	2021.10.5	Internal system correction	Qualified
7	2021.10.6	2021.10.10	System authorization	Qualified

## Data Availability

The data used to support the findings of this study are included within the article.
